# Genetic, Structural, Physicochemical, and Molecular Epidemiological Landscape of Three New Mutations Found in the Spike (S) Protein of Highly Transmissible Sri Lankan Delta Variant Sub-lineage AY.28: A222V, A701S, and A1078S

**DOI:** 10.1155/2022/4364131

**Published:** 2022-10-27

**Authors:** Dilantha Gunawardana

**Affiliations:** Research Council, The University of Sri Jayewardenepura, Gangodawila, Sri Lanka

## Abstract

Recently, three new mutations were identified in Sri Lanka in the spike protein of the rapidly spreading delta variant of the SARS-CoV-2 virus identified by the sublineage AY.28. They were A222V, A701S, and A1078S. The primary focus here is on the A701S mutation that is (1) found in the immediate vicinity of the S1/S2 cleavage site (PRRAR*∗*SV) that separates S1 and S2 subunits of the spike protein; (2) has high structural disorder of the region spanning Serine-701 (Ser-701), which promotes a longer flexible loop forming a better substrate; (3) collapses a loose, short, unstable, tripeptide beta strand (ENS), which is likely to assist the host proteases to cleave the S1-S2 interface easily than when an alanine is present. The same A701S mutation is found in at least 10 other strains of SARS-CoV-2 found in India, USA (East and West Coasts), and China, which classifies this mutation as geographically widespread and convergent in etiology. Conversely, the A1078S mutation is a highly present (>60 strains) mutation in terms of the SARS-CoV-2 coronaviruses, while the highly abundant A222V mutation is inferred by the genetic code, structural and topological features, and placement (in a beta strand) to be an innocuous, conservative mutation. The critical nature of S1/S2-dependent cleavage of S1 and S2 subunits of the spike protein makes the A701S mutation one of significance not just for possible higher virus transmission but also for subsequent fates such as viral load and vaccine effectivity against the delta variant.

## 1. Introduction

A pandemic (COVID-19) set in motion by the SARS-CoV-2 (severe acute respiratory syndrome) coronaviruses, types of positive sense RNA viruses, belonging to the beta coronavirus family, have engulfed our planet which until the 20^th^ of August 2021, has claimed 4,421,380 human lives and has resulted in high numbers of infections all over the world [1]. In Sri Lanka, the number of deaths has gone past 6500 as of the present. There are members of the coronavirus family that are benign, such as 229E, NL63, OC43, and HKU1, only provisioning mild symptoms, while conversely, three coronaviruses, SARS-CoV, MERS-CoV, and SARS-CoV-2, are deadly, with fatality rates of 10%, 37%, and 5%, respectively, to the host [2]. The delta variant of the SARS-CoV-2 had colonized every corner of the world in 2021 but was replaced by the omicron variant. In the arsenal of mutations of a key protein called the spike glycoprotein that the World Health Organization has classified the delta variant with, there is one that is of concern to the author (D614G), which is found not far from a mutation from this study (A701S), and is known to enhance the infectivity and titers of SARS-CoV-2 and is identified as the predominant form of the delta variant [3].

A key protein for a coronavirus to internalize into a receptive host cell is the spike protein which is made of two halves/subunits S1 and S2 [4]. The cells infected by the SARS-CoV-2 include basal-, ciliated-, club-, and AT2 cells in the lungs [5]. The SARS-CoV-2 forms a binding interface with the angiotensin converting enzyme-2 (ACE-2) receptor through the receptor binding domain (RBD) of the S1 subunit of the spike protein, thereby furnishing the binding of a receptor to a trimer, with a dissociation constant (*K*_*D*_) of ∼14.7 nM for the human-infective SARS-CoV-2 [2]. Out of lung cell types, ciliated-, club- and goblet cells, as well as AT2 cells, possess the ACE-2 receptors, while there are no reports of a significant presence of ACE-2 receptors in basal cells [5].

Most western and eastern nations have experienced multiple waves of the pandemic and a global vaccination drive is now quelling the sheer numbers in morbidities and mortalities of the SARS-CoV-2 virus. However, the nature of new mutations that are harmful for the host have resulted in unforeseen horizons, troubling both recipient cells of the human lungs, as well as well-organized health systems of developed nations. SARS-CoV-2 coronaviruses were thought to originate from Wuhan, China (Hubei Province), and is hypothesized to have crossed the zoonotic barrier from bats to humans [6]. The ability of the SARS-CoV-2 coronaviruses to mutate in spite of having a proofreading effector in nsp14 (nonstructural protein 14/exonuclease) does bring to the spotlight the RNA-dependent RNA polymerase that should be rather erroneous in execution of its routine functions [7].

Mutations come in an array of forms, and primarily as single nucleotide substitutions (nonsense/missense/synonymous, etc). In such a landscape, the alterations in genetic code coding for the amino acids are crucial for the surveillance efforts of the virus. Amino acids number to 20 and are the building blocks of cellular proteins. Amino acids can be classified by physicochemical structures, as well as by their encoding codons that are given three letters of the RNA alphabet. In this *in silico* research article, three mutations (A222V, A701S, and A1078S) in the delta variant of SARS-CoV-2 identified in Sri Lanka are forensically studied to showcase one mutation (A701S) that is inferred by the author as a crucial one for the host proteases to cleave the spike protein (at the S1-S2 interface) of the virus into two unequal parts that are functional for (1) the activation/promotion of receptor binding by the RBD of S1 subunit and (2) internalization of the virus into the host cells, respectively.

A mutation can be elucidated by its distance in the genetic code, the polar topological spaces the two amino acids utilize, the physicochemical attributes of sidechains, and structure-function relationships that are arrived upon by the secondary structure, amino acid type, and the convergency of the mutation as a favorable change [8]. Therefore, this study in summary is a bioinformatics exploration on the potency of the three recently recorded mutations in the spike protein of SARS-CoV-2 and how it is likely to impact human health in Sri Lanka.

## 2. Results and Discussion

### 2.1. Genetic Perspective

Serine is the most frequently found mutation and one of the most targeted destinations in relation to amino acids and consequently, is called a mutational hotspot [8]. This is primarily due to the two disjointed types of codons that are found in the genetic code that are encoding for the same amino acid, serene [9]. They are as follows: UCN (UCA, UCC, UCG, and UCU) and AGY (AGU and AGC), which are farther apart than a single nucleotide substitution, which makes two distant groupings and six unique codons for serine (Figure 1). The A701S and A1078S mutations are found in the S2 part of the spike protein and located within two linker regions: one between RBD and FP and the other between HR1 and HR2 (Figure 2). The change of an alanine to a serine can be effectuated in two ways.

1. For UCN (UCA, UCC, UCG, and UCU) codons of serine: single nucleotide changes at position 1 of all codons of alanine to become serines
2. For AGY (AGU and AGC) codons of serine: a minimum two sequential changes from the 4 codons of alanine, to arrive at serine.

On the other hand, the A222V mutation, a nonsynonymous substitution type, appears to be a single nucleotide change at the second position of all four alanine codons.

### 2.2. Structural Perspective

#### 2.2.1. A701S Mutation

Ala-701 and Ala-1078 are largely conserved between SARS-2 type pangolin and bat coronaviruses (Figure 2). Only at position 701 in the SARS-like coronavirus BatCoV/BB9904/BGR/2008, the alanine is mutated to a glutamate (E), which is a negatively charged amino acid. The A701S mutation is found in close proximity to the S1/S2 cleavage site (PRRAR*∗*SV sequence) in the human SARS-CoV-2- coronaviruses (Figure 2) and may have a potent role in the reactive footprint of binding of the proteases for the subsequent cleavage of S1 and S2 subunits. There are also two glycosyl sites that are immediately C-terminal (20–30 residues downstream) to the Ser-701 in the S2 protein sequence of SARS-CoV-2 viruses (Figure 2). Since the surface-exposed area of the S1/S2 cleavage site is made of a loosely disordered region, it was decided to assess the overall structural disorder in this important region surrounding the protease cleavage site using the PSIPRED workbench. Although the structural disorder was not >0.5 (cut off threshold) (Figure 3), the region spanning the S1/S2 cleavage site has a strong structurally disordered region that spans from ∼670 to ∼710 amino acids of the respective sequence.

The adjacent sequence surrounding the S1/S2 cleavage site was explored using a 38 residue stretch on either side of the S1/S2 protease cleaving site **(N-terminal (671)—ASYQTQTNSPRRARSVASQSIIAYTMSLGSENSVAYSN-C terminal (709))**, when many spike protein sequences with an identical S701A mutation were discovered in China (1), India (1), and the USA (both East and West Coast) (8) (Table 1). Therefore, 10 other viral strains (from diverse parts of the world) contain the same mutation (A701S) as the Sri Lankan variant. This suggests that this mutation may be an important one, both from its location/locality and its involvement in the S1/S2-dependent cleavage potential of the substrate polypeptide. Furthermore, 37/38 residues being identical in all 10 sequences show the recalcitrance of the region to mutation with the exception of the A701S mutation. Again, alanine is highly mutable and serine is a preferred mutational destination [8].

When the structure of the native coronavirus strain (SARS-CoV-2) without the S701A mutation is visualized in 3-D, it can be clearly seen that the A701S mutation can collapse a fragile tripeptide (ENS) into a significantly longer loop structure (Figure 4). This random coil loop is found near the end of a longer span containing the S1/S2 cleavage site that has a structurally disordered region (Figure 4). Therefore, it is predicted here that the tripeptide beat sheet (ENS) will collapse/loosen to form a longer more flexible loop region, contributing to the virus's potency or facilitate in its cleavage of the spike protein into separate S1 and S2 parts. A longer dangling loop will be more prone to better fit into the substrate binding site of the host protease and be cleaved.

Furthermore, the order of the commonest amino acids in loops connecting beta strands is Asn > Gly > Asp > Ser > Thr, which further strengthens the argument presented by the author here, due to serine being the fourth commonest amino acid in between beta strands [10]. Loops have many biological functions such as recognition of incoming molecules (example, antibodies), ligand binding and in the induced-fit anatomy (of substrate loops) for enzyme binding sites in serine, and other proteases [10]. As shown in Figure 6(a), the loop region where Ala-701 is found is surface-exposed (open for interactions with incoming macromolecules) and forms a lengthy, loosely disordered thread of amino acids interrupted by a short ENS beta strand, which I infer to collapse due to the A701S mutation.

It is of note that the D614G mutation which is the signature mutation for the dominant delta variant is only found 35 amino acids N-terminal to the structurally disordered (∼650–710) region of the S1-S2 junction of the spike glycoprotein and both mutations together can play a combined role for higher infectivity and higher titers, which could be detrimental to the magnitude of COVID-19 in patients infected with a strain harboring the twin mutations. There are also records that the delta variant has attenuated sensitivity to antibody neutralization, which also can have repercussions for vaccine efficacy [11].

#### 2.2.2. A1078S Mutation

The A1078S mutation when scrutinized was found in between the HR1 and HR2 sequences that form a dimerization interface; therefore, this mutation may too be one of crucial etiology for a positively impacting function in viral biology. Therefore, I searched the whole sequence of the S2 protein (including the C-terminal moiety of S1) to identify the secondary structural motifs that are prevalent in this structure (Figure 5), which showed an unknown localization or being present in the cytoplasm. The position of the Ala-1078 between two beta strands and the flexibility of a single proline between two alanine (sequence of Ala-Pro-Ala) is bound to be key to the positioning of the alanine and the A1078S mutation is again capable of forming a longer loop which may have rewired functions depending on hydrogen bonds and other molecular interactions. Furthermore, the mutation A1078S was found in numerous (>60) SARS-CoV-2 coronavirus strains when searched using the BLASTp tool. Therefore, the sheer number of positive hits prevents the tabulation of the details of specific geographical locality of this particular mutation, as performed for the A701S mutation.

#### 2.2.3. A222V Mutation

A222V mutation, a conservative nonsynonymous substitution type, is found inside a beta strand (Figure 6(b)), which is in agreement with the nature of the donor and recipient mutable species, as hydrophobic residues. Therefore, this mutation is unlikely to impact the viral biology significantly.

### 2.3. Physicochemical Perspective

The physicochemical features of serine are well suited for minimum obstructions and maximum slippage to protein features that are crucial for structure-function relationships. The side chains of serine are not bulky (Figure 7(a)) and therefore pose minimal steric and functional restrictions to immediately neighboring amino acids, as well as those in close proximity in space but not in sequence. Therefore, on top of the 6-codon coverage of the amino acid serine, it is also compliant for many kinds of polar surfaces and this property makes serine a frequent mutation (a mutational hotspot) that can undergo natural selection.

While for the physicochemical properties of an alanine to valine mutation (A222V), the exchange of a single hydrophobic residue for yet another hydrophobic residue, which according to the principles of biochemistry, suggests a rather innocuous modification. This mutation will not be studied in strong detail here. Valine and alanine have the same topological polar surface area of 63.3 A^2^, with only an extra methyl group placed in the structure of valine [Figure 7(B) and 7(C)].

### 2.4. Molecular Epidemiology

Molecular epidemiology of the delta variant in Sri Lanka can be inferred by sequencing of SARS-CoV-2 genomes. Three mutations, A222V (92.80%), A701S (88.06%), and A1078S (92.04%), were classified as lineage specific mutations in the AY.28 sublineage [12]. The authors of the abovementioned preprint suggests a fitness superiority of the AY.28 sublineage of the delta variant, over the co-occurring strains, which are identified as B.1.617.2 (parental) and AY.104 (sibling strain). Here, the fitness advantage of AY.28 is attributed to the A222V mutation, which is the second most prevalent substitution in the spike protein and is known to be benign on the virus phenotype [12]. The elevated presence of the A222V mutation is attributed to luck than to a selective advantage. However, there is evidence against this scientific theory of fortitude; that the background parental D614G mutant clade is improved in virulence, albeit slightly, by the A222V mutation [13].

In my study, I attribute the dominant transmissibility of the AY.28 version of the delta variant in Sri Lanka to the A701S mutation. A conservative mutation, A701V, has been shown to occur in the N501Y variant [14] that is known to produce more viral titers and to enhance viral replication and transmission. The same A701V mutation is attributed as improving the flexibility of the spike glycoprotein for better receptor binding, which agrees with the author's analyses here. However, the abovementioned mutation (A701V) substitutes a parental alanine with a similarly hydrophobic valine and does not replace the alanine with a polar serine, as is the case in the AY.28 strain. Still, the A701V mutation has been identified as a predominant mutation (in addition to D614G) in the widely circulating the SARS-CoV-2 strain B.1.524 in Malaysia and has been attributed a higher fitness compared to strains lacking the above mutation [15].

From the Colombo district (Sri Lanka) itself during the time period of July 2021 to October 2021, AY.28 was responsible for 57% of the delta genomes sequenced, while the other two strains, derived (AY.104) and parental (B.1.617.2), were found at 24.8% and 8% occurrence frequencies [12]. Therefore, molecular epidemiology suggests that one, two, or all three of the mutations, A222V, A701S, and A1078S, as providing a fitness advantage (in transmission) above the parental strain, B.1.617.2. Structural biology performed in this study attributes this advantage to the A701S mutation. At the pinnacle of the delta variant (August to September 2021), AY.28 sublineage was responsible for 128/189 (67.7%) of the infections, showcasing again the heightened virulence of the strain in concern [12]. As for disease severity, AY.28 sublineage is sublethal with only 3/160 developing mid-severe illness with one individual succumbing to the strain, while there were no deaths in the derived sibling (AY.104) and parental (B.1.617.2) strains [12]. Such mortalities and severe disease conditions in a minority can be due to a particular mutation's interaction with the genetic landscape and to the noncommunicable disease portfolios of the person in question as well as biochemical factors, such as cross-reactivities with natural and synthetic chemicals.

Furthermore, ORF3a coding for the largest protein of SARS-CoV-2 that includes a papain-like protease domain showed a significantly higher sgRNA expression in AY.28 in direct comparison to AY.104 (*p* < 0.0001) [12]. ORF3a is a polymorphic protein that possesses multifunctionality and is known to continually evolve similarly to the spike protein [16]. Therefore, the higher expression of ORF3a can be inferred to play a role in its higher involvement in virulence of AY.28 strain.

## 3. Conclusions

In this study, the three most recent mutations identified in the Sri Lankan form of the easily transmitted delta variant of SARS-CoV-2 (AY.28) are analyzed and genetic, structural, and physicochemical analyses were performed, to ascertain *in silico* what the mutations mean to viral function and human health. In particular, the A701S mutation appears likely to alter the S1/S2 protease cleavage site function by enhancing the flexibility of the loopy protein substrate by the likely-collapse of a poorly formed, unstable, and short beta strand of the spike protein. This is likely to improve the infectivity of the delta variant by accommodating more flexible binding of the loopy substrate by the host proteases and may have repercussion on viral loads and vaccine efficacy. The A701S mutation is found as a rare modification within the S1-S2 junction region in 10 strains of SARS-CoV-2 from independent localities including USA, China, and India, which can impact future fates in a pandemic hit world. Finally, molecular epidemiology numbers attribute the three AY.28 sublineage specific mutations as the reason for the dominance of this strain compared to the parental and sibling strains in Sri Lanka.

## 4. Methods

### 4.1. BLAST and Protein Search Tools

The BLASTp search tool [17] was used for the identification of mutations found all over the world to ascertain the availability of such changes. Sequences spanning the functional areas (example: S1/S2 cleavage site) were used with a substitution mutation (changing A to S) prior to running the search. The NCBI protein database was used for word-based searches of the spike proteins from humans.

### 4.2. Protein Structural Disorder and Secondary Structure Prediction

Protein structural disorder prediction and secondary structural features discovery were performed using the PsiPred workbench [18].

### 4.3. Protein 3-D Structure Visualization

Protein structures were visualized from the sequence repositories of the Protein Data Bank (PDB) using the Mol*∗* 3D Viewer [19].

### 4.4. Topological Polar Surface Areas Determination

Topological polar surface areas of each amino acid were obtained from PubChem [20].

## Figures and Tables

**Figure 1:** The genetic code of mRNA arranged as nucleotide triplets making up the identity of the codons. The link can be found at https://commons.wikimedia.org/wiki/File:Genetic_Code.png.

**Figure 2:** Sequence alignment of spike glycoprotein of selective coronaviruses. Link: https://www.ncbi.nlm.nih.gov/Structure/cdd/cd22378. In the figure, the domains of the S2 subunit of the spike protein of SARS-2 coronaviruses are shown. RBD–Receptor Binding Domain, HR1 and HR2—Heptad Repeats; FP-fusion peptide.

**Figure 3:** The structural disorder prediction of the sequence of the S protein (GenBank: QJX68370.1) using DISOPRED tool.

**Figure 4:** The zoomed structural views of Ala-701 (in pink) which is found prior to the commencement of a short betasheet ESN (structure shown is PDB ID: 6XCN). Alanine is predominantly found in beta strands but serine is primarily available in alpha helices [8]; consequently, the mutation A701S will destabilize the incumbent three residue beta strand and donate an extra residue for the structurally disordered loop. This mutation can collapse the beta strand into a longer coil structure and give flexibility to the S1/S2 protease susceptible region. This is further emphasized in the secondary structural prediction (Figure 5) where the tripeptide ENS is missing as a beta strand showing the instability of the region.

**Figure 5:** The secondary structural elements of the full-length SARS-2-CoV-2 predicted using the PSIPRED workbench.

**Figure 6:** (a) The position of the A701S mutation in the overall three-dimensional structure of the spike glycoprotein forming a surface-exposed, long, and flexible loop. (b) The placement of the alanine residue (pink/Ala-222) at the start of a beta strand.

**Figure 7:** (a) Structure of the amino acid, serine. (b) Structure of the amino acid, alanine. (c) Structure of the amino acid, valine.

**Table 1:** The 38 amino acid sequence containing a single mutation (A701S) was searched using BLASTp search tool to identify candidates containing the abovementioned mutation. The resulting 10 polypeptides tabulated below possess the A701S mutation and the remaining 37/38 residues were identical in sequence.

Sequence ID	Location
GenBank: QOS50451.1	India
GenBank: QPZ33389.1	China
GenBank: QWF04946.1	USA (Georgia)
GenBank: QYM28740.1	USA (California)
GenBank: QRK18727.1	USA (Georgia)
GenBank: QXG57847.1	USA (California)
GenBank: QXE65823.1	USA (Massachusetts)
GenBank: QWB84984.1	USA (Georgia)
GenBank: QTN61718.1	USA (Georgia)
GenBank: QUV65895.1	USA (Washington)

## Data Availability

Relevant data will be made available upon request.
